RETRACTED

# Immune landscape of periodontitis unveils alterations of infiltrating immunocytes and molecular networks-aggregating into an interactive web-tool for periodontitis related immune analysis and visualization

**DOI:** 10.1186/s12967-020-02616-1

**Published:** 2020-11-18

**Authors:** Xiaoqi Zhang, Qingxuan Wang, Xinyu Yan, Yue Shan, Lu Xing, Minqi Li, Hu Long, Wenli Lai

**Affiliations:** 1 Department of Orthodontics, State Key Laboratory of Oral Diseases, National Clinical Research Center of Oral Diseases, West China Hospital of Stomatology, Sichuan University, 14, Sect 3, Renmin South Rd, Chengdu, 610041 Sichuan China; 2 Department of Bone Metabolism, Shandong Key Laboratory of Oral Tissue Regeneration, School/Hospital of Stomatology, Shandong University, Jinan, Shandong, China

**Keywords:** Periodontitis, Immune, Immunocyte, Gene, Pathway, Web-tool, Bioinformatics

## Abstract

**Background:**

Immunity reaction plays an essential role in periodontitis progress and we aim to investigate the underlying regulatory network of immune reactions in periodontitis.

**Methods:**

CIBERSORT was used to estimate immunocyte fractions in different clinical statuses. Logistic regression was used to assess the immunocyte weight in periodontitis. Immune-related periodontitis subtypes were identified by the Nonnegative Matrix Factorization algorithm. Gene-set enrichment analysis and Gene-set variation analysis were conducted to analyze pathway activities. Immunocytes related gene modules were identified by Weighted gene co-expression network analysis.

**Results:**

Altered immunocytes in healthy versus periodontitis, aggressive versus chronic, male versus female and age were identified. Immunocytes enriched in periodontitis were calculated, and their correlation was also explored. Two distinct immune-related periodontitis subtypes were identified and one is characterized by B cell reactions and the other is IL-6 cytokine reactions. 463 statistically significant correlations between 22 immunocytes and pathways were revealed. Immunocytes and clinical phenotypes matched their gene modules, and their functions were annotated. Last, an easy-to-use and user-friendly interactive web-tool were developed for periodontitis related immune analysis and visualization (https://118.24.100.193:3838/tool-PIA/).

**Conclusions:**

This study systematically investigated periodontitis immune atlas and caught a glimpse of the underlying mechanism of periodontitis from gene-pathway-immunocyte networks, which can not only inspire researchers but also help them in periodontitis related immune researches.

## Background

Periodontitis is one of the three most common oral diseases with a high morbidity rate [1]. Epidemiological investigation revealed that periodontitis is the primary cause of tooth loss worldwide [2]. Periodontitis is characterized by the inflammatory destruction of periodontal support tissues, with main clinical manifestations including gingival inflammation, bleeding, periodontal pocket formation, alveolar bone resorption, progressive loss of attachment and tooth loosening and displacement [3]. Bacteria and their products in the plaque biofilm attached to and around the tooth surface can not only directly cause the inflammation and destruction of periodontal supporting tissues, but also trigger the host's immune and inflammatory response [4]. The progression of the disease not only depends on bacteria but also the host's immune response since the inappropriate immune response to microorganisms can accelerate the development and progress of periodontitis [5]. Therefore, host immune response, especially the immunocyte reaction, plays a key role in the balance between periodontal tissue repair and destruction. A lot of previous studies have demonstrated both innate and adaptive immunocyte reactions play an essential role in periodontitis progress such as dendritic cell [6], macrophage [7], neutrophil [8] in innate immunity responses, and CD4 T cells [9], CD8 T cell [10], and B cell [11] in adaptive immunity response. Hence, how immunocytes mediate the occurrence and development of periodontal inflammation and alveolar bone destruction and how the molecular regulation network function in immunocytes reaction and differentiation are the focus of current research on periodontitis.

RETRACTED

Nowadays, we have been in the post-genome era and the cost of high-throughput sequencing is getting lower. This results in the generation of tens of thousands of high-throughput data. How to use bioinformatics to analyze and to make use of these data to the fullest is now the emerging challenge. High-throughput data were widely used in various fields including periodontitis. Yuko et al. used methylation array to identify periodontal disease-related methylation sites [12], Nisha et al. [13] used miRNA array detecting miR143-3p as a novel salivary biomarker for chronic periodontitis, and M et al. used gene array identifying distinct periodontitis subtypes [14]. However, in these studies high-throughput data were not fully used, only routine analysis has been performed and only a little useful information was generated from the numerous results. Besides, analyzing and interpreting these high-throughput data requires knowledge in bioinformatics and programming. Therefore, it is imperative to assist researchers by comprehensively analyzing these public data using advanced algorithmic systematically to find more research targets and to present the results in a simple form to researchers who are not familiar with bioinformatics.

RETRACTED

In this study, we aim to use several advanced bioinformatic methods to analyze the periodontitis related immunocytes from public data in multiple levels and aggregate the results as an interactive web-tool for periodontitis related immune analysis and visualization. As a result, genes, pathways and immunocytes alterations and relationships in periodontitis were systematically revealed and abundant discoveries were presented. Furthermore, a web tool was constructed. These can not only inspire researchers but also help them in periodontitis-related immune researches.

## Methods

### Data acquisition and process

The data used in this study was in GSE16134 from the GEO (Gene Expression Omnibus) database [https://www.ncbi.nlm.nih.gov/geo/query/acc.cgi?acc=gse16134]. It contains expression data of 69 healthy samples and 241 periodontitis samples. The detailed information was described in the previous studies [14]. The raw data preprocesses were performed according to the standard procedure for Affymetrix microarray and prepared data for the CIBERSORT algorithm. The clinical information was obtained from Prof. P.N. Papapanou from Columbia University by personal communication on 7/25/2019.

### Bioinformatic analysis

CIBERSORT was used to estimate the proportion of infiltrating immunocyte subsets by transforming gene expression matrix to 22 types of immunocyte fractions matrix [15]. The immune-related gene list was obtained from the ImmPort database [https://www.immport.org]. Differentially expressed gene (DEG) analysis was performed by R package “limma”, and was conducted according to its pipeline, which is described before [16]. Genes with |logFC|> 1 and FDR < 0.01 were regarded as DEGs in periodontitis. The protein–protein interaction (PPI) network was conducted from the STRING database [https://string-db.org/] and beautified by CytoScape. The Gene Ontology and KEGG function enrichment analysis and GSEA (Gene-Set Enrichment Analysis) were performed using the R package “clusterProfiler”. GSVA (Gene Set Variation Analysis) was conducted using the R package “gsva”, which transforms an expression matrix to the gene-set score matrix. The R package “NMF” was used for consensus molecular subtyping [17]. The optimal number of subtypes was selected according to cophenetic, dispersion, and silhouette coefficients [18]. WGCNA (Weighted gene co-expression network analysis) analysis was conducted by R package “WGCNA”. The top 25% of genes with the largest variation were included and samples far from the main cluster were excluded. The analysis processes of WGCNA were described in detail in a previous study [19–21].

RETRACTED

### Statistical analysis and visualization

Samples with a CIBERSORT P value of <0.05 were included in the analysis. R software 3.6.1 was conducted in this study for the statistical analyses and visualization. R package “ggplot2”, “ggpuber” were used to make statistical plots including bar-plots, box-plots, violin-plots volcano-plots, and scatter-plots. R package “pheatmap” was used for heatmaps. The periodontitis related immunocytes and immune genes were identified by univariate logistic analysis. LASSO (Least absolute shrinkage and selection operator) regression was used for dimension reduction in immunocytes. Multivariate logistic regression was used to identify immunocytes related to periodontitis independently. For differences of immunocyte fractions between different clinical groups were analyzed by a two-sided Wilcoxon rank-sum test. Correlation analysis was performed using the Spearman test. The P value was adjusted by the FDR method for multiple hypothesis testing. Dichotomous variables were compared using the chi-square test. The web-tool was constructed by R package “shiny”.

## Results

### Infiltrating immunocytes landscape in periodontitis

To explore the differences of infiltrating immunocytes between healthy and periodontitis tissues, CIBERSORT algorithm was conducted to reveal the distribution of 22 immunocyte fractions and we found no matter in healthy or periodontitis tissue the plasma cells took up the largest fraction (Fig. 1a). We compared the fractions of 22 immunocytes between healthy and periodontitis, and 13 immunocytes were altered in periodontitis tissue including 5 increasing immunocytes fractions (plasma cell, neutrophils, T cells CD4 memory activated, dendritic cells activated and NK cells resting) and 8 decreasing immunocytes fractions (Tregs, dendritic cells resting, eosinophils, mast cells resting, macrophages M1, B cells memory, T cells follicular helper and T cells CD4 memory resting) in periodontitis tissue (Fig. 1b, Additional file 1: Table S1). The most downregulated and upregulated immunocytes are Tregs and neutrophils, respectively (Fig. 1c). Then, to explore if the variation in immunocytes proportions could be an intrinsic feature that may characterize the individual diversities, we performed PCA analysis and found that the proportions of immune cells displayed distinct clustering and individual differences (Fig. 1d). Among them, plasma cells, B cell memory and mast cells resting contributed the most in the healthy and periodontitis tissue variation. Correlation analysis was performed in periodontitis samples and all samples. We found in both periodontitis and all samples that B cell memory and plasma cells were the most negatively correlated, to plasma cells and macrophages M1 (Fig. 1e). Further, the differences of infiltrating immunocytes in different clinical subgroups were also investigated including periodontitis subtype, gender, and age by using similar analysis strategies (Additional file 2: Figure S1).

RETRACTED

**Fig. 1:** Infiltrating immunocytes differences between healthy and periodontitis samples. **a** The relative fraction of immunocytes identified by the CIBERSORT algorithm, which estimates relative subsets of 22 types of immunocyte from known RNA transcripts. The relative distributions of these 22 immunocytes were presented by bar-plots concerning different disease status (all samples for the left and average for the right). **b** Compositional differences of 22 immunocytes between healthy and periodontitis presented by violin-plot (blue means healthy and red means periodontitis). **c** The volcano-plot demonstrates the fold changes of 22 immunocytes in periodontitis compared with healthy. **d** Principal component analysis (PCA) of 22 infiltrating immunocytes between healthy and periodontitis. The two first principal components (PC1, PC2) which explain the most of the variables are plotted. **e** Correlation matrix of 22 immunocytes proportions. The top right is correlations of 22 immunocytes in all samples and the left bottom is correlations of 22 immunocytes in periodontitis samples

To explore and identify the robustness and contributing weight of immunocytes that are related to periodontitis independently, we conducted a series of regression algorithms to adjust the immunocyte interaction effect including univariate logistic regression, LASSO regression, and multivariate logistic regression. 12 periodontitis-related immunocytes were first identified by univariate analysis (Fig. 2a). Then, LASSO regression was performed to make feature selection and dimension reduction so that the unimportant immunocytes could be excluded. Therefore, we screen out 11 important periodontitis-related immunocytes through LASSO regression (Additional file 2: Figure S2). Last, multivariate logistic regression was conducted on the 11 immunocytes evaluate their independency. Only the dendritic cells resting, dendritic cells activated and T cells follicular helper were independently related to periodontitis (Fig. 2b).

**Fig. 2:** Periodontitis associations of immunocytes. **a** Forest-plot demonstrates associations between different immunocyte subsets and periodontitis by univariate logistic regression. **b** Forest-plot demonstrates the independent associations between periodontitis-related immunocytes and periodontitis by multivariate logistic regression

RETRACTED

#### Identification of immune-related periodontitis subtypes and their characteristics

To identify immune-related periodontitis subtypes, 1214 immune-related genes were compiled, and 702 of them were significantly related to periodontitis (FDR < 0.05) (Additional file 3: Table S2). Using the 702-gene panel, 2 distinct immune-related periodontitis subtypes were identified by performing consensus clustering analysis (Fig. 3a, Additional file 2: Figure S3A-C). Then, 116 genes were selected from all 702 immune-related genes and the sparse structure of the metagenes appeared in the localized patterns of the gene contributions, in which the 116 genes were defined as hub genes for each subtype representing the subtype characteristics (Fig. 3b, Additional file 2: Figure S3D). There were 45 immune-related genes representing subtype 1 (cluster 1) and 71 genes for subtype 2 (cluster 2). To get a further understanding of the regulation effects among these genes, the PPI networks of the 116 hub genes revealed their relationships and importance in the network., in which CXCR4 of cluster-1 has the most links with other genes and PIK3RI in cluster-2 has the most (Fig. 3c, Additional file 4: Table S3).

**Fig. 3:** Identification of immune subtypes of periodontitis by consensus clustering. **a** The consensus matrix was obtained from 200 random runs of the Brunet et al.'s algorithm. Values range from 0 to 1. Columns and rows were ordered by hierarchical clustering based on the euclidean distance with average linkage. **b** Heatmap of the metagene matrix. Each row corresponds to a gene. The most metagene-specific genes were selected using Kim and Park's scoring and filtering methods. This resulted in the selection of 116 genes. Rows were scaled to sum to one and ordered by hierarchical clustering based on the euclidean distance and average linkage. **c** The protein–protein interaction network of 116 metagenes. The blue is immune subtype cluster-1 and red is subtype cluster-2. Only the genes with interaction with others are presented

To understand the characteristics and differences between the two immune-related subtypes, GO enrichment analysis and canonical pathway enrichment analysis was performed. Biological processes of GO were conducted and to simplify the results, we grouped categories according to the functional theme, which represents the biological characteristics of the cluster (Fig. 4a). The characteristics of cluster-1 were mainly concerning with FC-receptor and immune-associated receptor-mediated immune regulations such as FC/FC-gamma receptor signaling pathway and cell surface receptors. Another feature of cluster-1 is involved in B cell immune processes regulations such as B cell differentiation and B cell activation. As for cluster-2, the IL-6 cytokine feature is predominant such as regulation of IL-production. Then, canonical pathway analysis revealed the significantly enriched or activated pathways in cluster-1 and cluster-2 (Fig. 4b, c), which were in consistent with the results above, and we found some famous pathways were shown such as JAK-STAT signaling in cluster-1 and PK3K-AKT in cluster-2.

RETRACTED

**Fig. 4:** Functions and biological characteristics of immune subtypes. **a** The gene ontology enrichment analysis for the metagenes in two immune subtypes concerning their biological processes. GO categories are grouped according to functional. **b**, **c** The KEGG pathway enrichment analysis for the metagenes in two immune subtypes respectively (**b** for cluster-1 and **c** for cluster-2)

### Associations between immune subtypes and immunocytes

To investigate the diversities between the two immune subtypes from cell level, the 22 infiltrating immunocyte fractions were compared and clinical features were also compared. From the results, the two immune subtypes demonstrated distinct profiles in infiltrating immunocytes, in which 13 immunocytes were different (Fig. 5a, b). Distinct infiltrating immunocyte abundances were found between the two clusters of immune periodontitis subtypes. Cluster-1 has more infiltration of activated dendritic cells, plasma cells and neutrophils compared to cluster-2. While for cluster-2, more B cell memory, T cells CD4 memory resting, T cells follicular helper, NK cells activated, monocytes, macrophages M1, macrophages M2, dendritic cells resting, mast cells activated and mast cells resting were upregulated compared with cluster-1. Besides, we noticed cluster-2 was significantly associated with chronic periodontitis and cluster-1 associated with aggressive periodontitis (Fig. 5c), while there is no different distribution between two clusters concerning gender and age.

**Fig. 5:** Correlations between immune subtypes and immunocytes. **a** Compositional differences of 22 immunocytes between immune subtype cluster 1 and cluster 2 which was presented by violin-plot (blue means cluster-1 and red means cluster-2). **b **Comparison of immune-related pathways’ activity between the two immune subtypes. **c** Comparing periodontitis subtypes, genders, and ages between immune subtype cluster 1 and cluster 2. The heatmap illustrates the association of different clinical characters with cluster 1 and cluster 2 patients. Statistical significance was performed by the χ^2^ test

RETRACTED

### Differentially expressed genes and gene-sets between healthy and periodontitis

To understand the molecular mechanisms by which genes or gene-sets drive the biological reactions in the periodontitis, DEGs analysis and gene-set enrichment analysis were conducted. Using the criterion of FDR < 0.01 and |logFC|> 1, 171 DEGs were identified and 134 of them were up-regulated in periodontitis while 37 of them were down-regulated. These up-regulated genes may be involved in the progress of periodontitis, and among them, the MZB1, TNFRSF17, and IGLL5 are the top three up-regulated genes. The interaction relationships among these genes were also investigated and were presented as a PPI network (Fig. 6a). According to outward traversal from a locally dense seed protein and vertex weighting by local neighborhood density, these DEGs were divided into several molecular complexes and were presented by different shapes. Besides, the top ten hub genes among these genes were also identified with the highest links to nodes, indicating they are in the core position of the network and played an essential role in the regulation of the network.

**Fig. 6:** Transcriptome differences between healthy and periodontitis. **a** The protein–protein interaction network of significantly differentially expressed genes between healthy and periodontitis. The node size means the absolute value of logFC, the node with yellow frame means the hub genes with a high connective degree in the network, the red nodes mean the genes up-regulated in periodontitis and blue nodes mean the genes down-regulated in periodontitis. **b**–**e** Gene-set enrichment analysis from four aspects (including immunologic signatures, hallmark gene sets, GO biological processes and canonical pathways) revealed the underlying biomolecular differences between healthy and periodontitis

Not only were the individual gene was investigated, but also gene-sets. We mainly focused on four aspects of gene-sets including immunologic signatures, hallmark gene sets, GO biological processes and canonical pathways. Results showed many enriched gene-sets in periodontitis were associated with immune processes or regulations (Fig. 6b–e) such as CD4 T CELL VS B CELL DOWN in immunologic signature, IL6 JAK STAT6 SIGNALING in hallmark, POSITIVE REGULATION OF B CELL DIFFERENTIATION in GO and T HEPLER PATHWAY in the canonical pathway. All these four aspects implied immune-related response is essential in periodontitis.

### Identification of infiltrating immunocytes related hallmark pathways

To further understand the molecular mechanisms by which hallmark pathways are involved in immunocyte content, we examined the correlation between the fractions of 22 immunocytes and the activity of 50 hallmark pathways. In total, 463 statistically significant correlations between 22 immunocytes and 50 hallmark pathways were observed. Both T cells CD4 naive and B cell memory had 24 negatively correlated signaling pathways, which is the most compared with other immunocytes. While Plasma cells had 21 positively correlated signaling pathways which is the most among all immunocytes. (Fig. 7a, Additonal file 5: Table S4). The links with high correlation coefficients were presented (Fig. 7b) such as dendritic cells resting is negatively correlated with hallmark coagulation with − 0.56 correlation and plasma cells are positively correlated with hallmark unfolded protein response with 0.57 correlation.

RETRACTED

**Fig. 7:** Correlations between 22 immunocytes fractions and activity of 50 important biological hallmark-related pathways. **a** The number of significant pathways is correlated with individual immunocyte. The upper panel is for positively correlated pathways, and the bottom panel is for negatively correlated pathways. **b** Network diagram demonstrating the correlation between immunocytes and pathways. Red represents a positive correlation, and blue represents a negative correlation. The size of the nodes corresponds to the number of links, and the thickness of the line represents the correlation coefficient

### Infiltrating immunocytes related gene module identified by WGCNA

To understand the molecular mechanisms of alteration in infiltrating immunocytes in detail, the genes or gene modules regulating immunocytes or affected by immunocytes need to be uncovered. Therefore, WGCNA, an advanced bioinformatic algorithm, was conducted to find clusters (modules) of highly correlated genes related to external sample characteristics (immunocytes fractions). It is usually used to find a cluster of genes related to some features. 13 was used as network topology for thresholding power considering its relatively mean connectivity power and balanced scale independence (Additional file 2: Figure S4A-B). Clustering of module eigengenes was performed in the top 25% variance 4329 genes and 27 modules were identified (Fig. 8a, b). Each module was constituted by those highly correlated genes, which have similar functions. Then, the relationship between immunocyte fractions and clinical features were calculated and visualized according to their significance in a heatmap (Fig. 8c). In another word, the gene modules related to an immunocyte were identified (Additional file 6: Table S5). For example, the turquoise module was positively correlated with plasma cells the most, as we can see from the heat map and scatter plot (Fig. 9a), This suggested the genes in the turquoise module is involved in the regulation of plasma cell population or affected by increased plasma cell fractions. And in another way, it means plasma cell-related genes were identified. The genes with high gene significance and module membership were the key genes in the turquoise module and their interaction relationships were presented in the PPI network so that we could locate the central genes according to links degree (Additional file 2: Figure S4C). From the network, we noticed BTK has the most links in the network and is considered a hub gene. GO analysis was also conducted to assess the biological functions of the turquoise module, and it was found these genes were involved in B cell regulation (Fig. 9b). This also indicated that our results were reliable from another perspective. Furthermore, a lot of new and unreported plasma cell-related genes were also found (Fig. 9c–e, Additional file 2: Figure S4D).

RETRACTED

**Fig. 8:** Identification of immunocytes and clinical characteristics related to gene modules. **a** The sample clustering was based on the expression data of all samples. The top 25% of variation genes were used for the analysis by WGCNA and outlier samples were excluded. **b** Gene dendrogram obtained by average linkage hierarchical clustering. The color row underneath the dendrogram shows the module assignment determined by the Dynamic Tree Cut, in which 27 modules were identified. **c** Heatmap of the correlation between module eigengenes and the immunocyte fractions

**Fig. 9:** Plasma cells related genes. **a** A scatterplot of gene significance (GS) for plasma cell fraction versus module membership (MM) in the turquoise module. GS and MM exhibit a very significant correlation, implying that hub genes of the turquoise module also tend to be highly correlated with plasma cell fraction. **b** GO enrichment analysis concerning biological processes revealed the functions of hub genes in the turquoise module. **c** The top ten hub genes in the turquoise module and their GS and MM were presented by bar-pot. **d**, **e** The most plasma cell fraction correlated with two genes was presented by a scatter plot

### An easy-to-use and user-friendly web-tool for periodontitis related immunity analysis

To help periodontitis researchers used the results described and to establish broad access to results in this work as well as other aspects of interest in periodontitis, we established an easy-to-use and user-friendly interactive web-tool for researchers working on periodontitis (https://118.24.100.193:3838/tool-PIA/). We named this platform as Periodontitis Immune Atlas (PIA). PIA provides 6 modules for users: “Genes”, “Pathways”, “WGCNA”, “Correlations”, “Immunocytes” and “Functions”, and all the results in these six modules can be downloaded for usage. The “Genes” module (Fig. 10a) provides the DEGs between healthy and periodontitis in several forms. Users can browse the DEG list in a table and sort them by the way they like. Besides, a gene list of immune-related genes with their category is also presented. The specific gene of interest can be visualized by volcano-plot or box-plot. Two genes’ correlation analysis are also provided. The “Pathways” module (Fig. 10b) allows users to inquire the activity score of specific pathways and presented them by box-plot. Three commonly used pathway sets were included (hallmarks, KEGG and GO-BP). The correlation between the two pathways can also be investigated. The “WGCNA” module (Fig. 10c) provides analysis for phenotype and gene module. Users can find gene modules related to interesting phenotypes and the gene modules function can also be investigated. In the “Correlation” module (Fig. 10d), users can fully explore the relationships among genes, pathways, and immunocytes. “Immunocytes” module (Fig. 10e) allows users to visualize the status of immunocytes in different clinical statuses and the correlation between two immunocytes is also included. The “Functions” module (Fig. 10f) provides GSEA analysis between different clinical status. Besides, single-gene GSEA can be used as a function predictor for a specific gene in periodontitis. All figures generated in this platform can be downloaded for further analysis and the query results are demonstrated in a comfortable form. The functions provided in the web-tool, which will be continuously updated, may serve as a guide for researchers interested in periodontitis related immunity.

RETRACTED

**Fig. 10:** Overview of Periodontitis Immune Atlas app

## Discussion

The immunocytes and immune reactions play a key role in periodontitis progress, and uncovering the underlying regulation network and mechanism is urgent. To well address the problem, we conducted several advanced bioinformatic methods to systematically analyze immunity in periodontitis from three aspects including genes, pathways and immunocytes. First, we used CIBERSORT to convert an expression matrix to the immunocytes fraction matrix. 22 infiltrating immunocyte fractions were analyzed between different clinical statuses. Then a series of statistical algorithms were conducted to estimate the immunocyte weight contributing to periodontitis and identify the independent immunocyte affecting periodontitis [22]. And we found dendritic cells activated, dendritic cells resting and T cells follicular helper may play an essential role in periodontitis [23]. The fractions of five immunocytes increased (plasma cell, neutrophils, T cells CD4 memory activated, dendritic cells activated and NK cells resting) and eight immunocytes fractions decreased (Tregs, dendritic cells resting, eosinophils, mast cells resting, macrophages M1, B cells memory, T cells follicular helper and T cells CD4 memory resting) in periodontitis samples. Plasma cells increased by 20.66% in periodontitis, suggesting its leading role in periodontitis lesions [24]. Following B cell memory, which was decreased by 7.21% compared with healthy samples [25]. The mast cells resting reduced 4.06% and dendritic cells resting reduced 3.27%, indicating an upregulation of their activated status. Neutrophils increased 1.85% in periodontitis and this is in accordance with the inflammation status of gingival tissue. T cells CD4 memory activated increased by 0.59% while T cells CD4 memory resting decreased 1.99%, which suggested T cells CD4 memory were activated in periodontitis. Second, we used immune-related genes that are closely related to periodontitis to perform unsupervised clustering by the NMF algorithm [14, 17]. And two distinct immune subtypes of periodontitis were identified with their molecular features. The subtypes were different from the currently accepted periodontitis classification, but their distinct molecular phenotypes represented diverse periodontitis-related immune characteristics. The identification of two immune periodontitis subtypes is based on the NMF algorithm. Nonnegative Matrix Factorization (NMF) is an unsupervised learning technique that has been applied successfully in several fields, including signal processing, face recognition and text mining. Recent applications of NMF in bioinformatics have demonstrated its ability to extract meaningful information from high-dimensional data such as gene expression microarrays [17]. From the results, more cases of chronic periodontitis were clustered in subtype-2 which is in accordance with its immune characteristics, in which IL-6 cytokine has been well characterized as a major player in chronic inflammation [26]. In aggressive periodontitis, infiltration ofCD4, CD8, CD20 and CD68 cells were observed. Likewise B cell immune processes were involved in cluster-1 which had more cases of aggressive periodontitis [27]. The results suggested that immune-related genes of periodontitis tissues can provide an alternative classification of periodontitis that is associated with immune characteristics [28], which enhanced the understanding of the immune pathobiology in periodontitis. Third, the GSVA algorithm was employed to convert the expression matrix to a pathway activity score matrix, so that the relationship between pathways and immunocytes can be unveiled [29]. Common pathways positively or negatively correlated to immunocytes were fully investigated, which implies these pathways may be involved in immunocytes regulation or affected by immunocytes. Pathways are the bridge between genes and immunocytes. Last, WGCNA was conducted to investigate the relationship between gene modules and phenotypes. Genes were grouped into modules according to their similarity and the correlation between gene module and phenotypes were investigated. For example, the turquoise module is significantly related to plasma cells fractions indicating genes of turquoise module may be involved in the regulation of plasma cells. This analysis revealed the relationship between genes and immunocytes. As far as we know, all the four aspects of analysis about periodontitis immune regulation were the first time to be conducted in our study. They systematically explained the periodontitis immune regulation network from gene-pathway-immunocyte.

RETRACTED

At present, there is a lack of such systematic and comprehensive bioinformatics analysis in the periodontal research, and there are few studies on immune cells using high-throughput data, and a huge amount of information hidden behind these data were left unexplored. However, in other fields, particularly oncology, bioinformatics analysis and the use of high-throughput data have become the norm [30, 31], which help researchers identify research targets and predict results. In our study, we a series of bioinformatic analysis were conducted from which abundant results were generated that couldinspire other researchers. To facilitate immune-related research in periodontitis, we developed the PIA (Periodontitis Immune Atlas) App, an easy-to-use and user-friendly web-tool for comprehensive analysis of gene, pathway and immunocyte data in periodontitis. The PIA App integrates several advanced bioinformatic methods and provided customized functions and interactive operation including gene-related analysis, pathway-related analysis, immunocytes-related analysis, WGCNA analysis, correlation analysis and functional analysis for users to explore the immune-related researches in a multi-dimensional manner. The PIA app serves as a new approach for users, especially wet-bench scientists with no programming background, to analyze the scientific big data and facilitate data mining [32]. It is an interactive web application, which enables experimental researchers without any computational programming background to perform multiple analyses related to periodontitis immunity. Using the PIA App, one can easily explore the large and systematical data, ask specific scientific questions, and validate their findings.

RETRACTED

We have to acknowledge that there are some shortcomings in our study. The dataset GSE16134 we analyzed was somewhat incomplete. Because the follow-up information, precise clinical classification and many other clinicopathological data were not provided, relevant analysis cannot be performed so that we weren’t able to find out if there were other distinct clinicopathological characteristics between the two immune periodontitis subtypes. Analyzing infiltrating immunocyte fractions using a machine learning algorithm from transcriptome data may not be the best way and single-cell sequencing should be the current best way to precisely analyze infiltrating immunocytes from a bulk tissue [33]. Still, before the emergence of single-cell sequencing data of periodontitis, CIBERSORT algorithm was the best approach to analyze infiltrating immunocytes we can use in periodontitis [34, 35]. Besides, considering the high cost and complex technology of single-cell sequencing, it would be a good thing to use such a simple and effective method to study immune infiltration in periodontitis before the popularization of single-cell sequencing, if the CIBERSORT can be verified experimentally with high accuracy. We believe this CIBERSORT is accurate enough, after all, it is widely used and verified in other fields [36–38]. Therefore, the results of this study deserve more attention.

## Conclusions

In conclusion, we systematically analyzed periodontitis infiltrating immunocytes alterations in different clinical status and identified several important immunocytes related to periodontitis by multiple methods, including dendritic cell resting, dendritic cell activated and T cell follicular helper. Two immune-related periodontitis subtypes were identified and the relation with immunocytes, clinical features and biological functions were investigated. Pathways associated with immunocyte fractions were revealed. Immunocytes related genes were also identified. These results caught a glimpse of the underlying mechanism of periodontitis from gene-pathway-immunocyte networks. Further, a web-tool for analyzing and visualizing periodontitis related immune was constructed (https://118.24.100.193:3838/tool-PIA/). These can not only inspire researchers but also help them in periodontitis-related immune researches.

## Supplementary information

**Additional file 1: Table S1.** The list of immunocyte difference between healthy and periodontitis samples.

**Additional file 2: Figure S1.** Infiltrating immunocytes differences. (A) The volcano-plot demonstrates the fold changes of 22 immunocytes in chronic periodontitis compared with aggressive. (B) Compositional differences of 22 immunocytes between chronic and aggressive periodontitis presented by violin-plot (blue means aggressive and red means chronic). (C) The volcano-plot demonstrates the fold changes of 22 immunocytes in male periodontitis compared with female. (D) Compositional differences of 22 immunocytes between male and female periodontitis presented by violin-plot (blue means male and red means female). (E) Correlations between infiltrating immunocyte fractions and patient ages were presented by bar-plot. (F-G) The two significantly age-related immunocytes were presented by scatter plot.** Figure S2.**(A) Least absolute shrinkage and selection operator (LASSO) coefficient profiles of 22 immunocytes fractions. The dotted line indicates the value chosen by ten-fold cross-validation. (B) Ten-fold cross-validation for tuning parameter selection in the LASSO regression. The partial likelihood deviance is plotted against log (λ), where λ is the tuning parameter. Partial likelihood deviance values are shown, with error bars representing SE. The dotted vertical lines are drawn at the optimal values by minimum criteria and 1-SE criteria. **Figure S3.** Supplementary information for immune subtype analysis. (A) Estimation of the rank: Quality measures computed from 200 runs for each value of r. (B) Estimation of the rank: Consensus matrices computed from 10 runs for each value of r. (C-D) Heatmap of the mixture coefficient and the basis matrices for all immune genes. **Figure S4.** Supplementary information for WGCNA analysis. (A) analysis of the scale-free ft index for various soft-thresholding powers beta. (B) Analysis of the mean connectivity for various soft-thresholding powers. (C) The protein-protein interaction network of hub genes in turquoise module. (D) The top ten positive and negative plasma cell fraction related genes, calculated by pearson correlation analysis.

RETRACTED

**Additional file 3: Table S2.** The list of univariate logistc regression analysis for immune genes related to periodontitis.

**Additional file 4: Table S3.** The list of cluster specific genes.

**Additional file 5: Table S4.** The list of correlation analysis between immunocytes and HALLMARK pathways.

**Additional file 6: Table S5** The list of WGCNA resutls.

## Data Availability

The datasets generated and analyzed during the current study are available in the GEO repository [https://www.ncbi.nlm.nih.gov/geo/].

## Abbreviations

WGCNA: Weighted gene co-expression network analysis
MM: Module membership
GS: Gene significance
GSEA: Gene-set enrichment analysis
GSVA: Gene-set variation analysis
GO: Gene Ontology
BP: Biological process
KEGG: Kyoto encyclopedia of genes and genomes
PCA: Principal component analysis
LASSO: Least absolute shrinkage and selection operator
DEG: Differentially expressed gene
PPI: Protein–protein interaction

## References

[1] Slots J (2000). Periodontitis: facts, fallacies and the future. Periodontol.

[2] Eke PI, Dye BA, Wei L, Slade GD, Thornton-Evans GO, Borgnakke WS, Taylor GW, Page RC, Beck JD, Genco RJ (2015). Update on prevalence of periodontitis in adults in the United States: NHANES 2009 to 2012. J Periodontol.

[3] Darveau RP (2010). Periodontitis: a polymicrobial disruption of host homeostasis. Nat Rev Microbiol.

[4] Hernandez M, Dutzan N, Garcia-Sesnich J, Abusleme L, Dezerega A, Silva N, Gonzalez FE, Vernal R, Sorsa T, Gamonal J (2011). Host-pathogen interactions in progressive chronic periodontitis. J Dent Res.

[5] Amano A (2000). Host-parasite interactions in periodontitis: microbial pathogenicity and innate immunity. Periodontol.

[6] Xiao W, Dong G, Pacios S, Alnammary M, Barger LA, Wang Y, Wu Y, Graves DT (2015). FOXO1 deletion reduces dendritic cell function and enhances susceptibility to periodontitis. Am J Pathol.

[7] Garaicoa-Pazmino C, Fretwurst T, Squarize CH, Berglundh T, Giannobile WV, Larsson L, Castilho RM (2019). Characterization of macrophage polarization in periodontal disease. J Clin Periodontol.

[8] White PC, Chicca IJ, Cooper PR, Milward MR, Chapple IL (2016). Neutrophil extracellular traps in periodontitis: a web of intrigue. J Dent Res.

[9] Hienz SA, Paliwal S, Ivanovski S (2015). Mechanisms of bone resorption in periodontitis. J Immunol Res.

[10] Cardoso EM, Arosa FA (2017). CD8(+) T cells in chronic periodontitis: roles and rules. Front Immunol.

[11] Zouali M (2017). The emerging roles of B cells as partners and targets in periodontitis. Autoimmunity.

[12] Kurushima Y, Tsai PC, Castillo-Fernandez J, Couto Alves A, El-Sayed Moustafa JS, Le Roy C, Spector TD, Ide M, Hughes FJ, Small KS (2019). Epigenetic findings in periodontitis in UK twins: a cross-sectional study. Clin Epigenetics.

[13] Nisha KJ, Janam P, Harshakumar K (2019). Identification of a novel salivary biomarker miR-143-3p for periodontal diagnosis: a proof of concept study. J Periodontol.

[14] Kebschull M, Demmer RT, Grun B, Guarnieri P, Pavlidis P, Papapanou PN (2014). Gingival tissue transcriptomes identify distinct periodontitis phenotypes. J Dent Res.

[15] Newman AM, Liu CL, Green MR, Gentles AJ, Feng W, Xu Y, Hoang CD, Diehn M, Alizadeh AA (2015). Robust enumeration of cell subsets from tissue expression profiles. Nat Methods.

[16] Ritchie ME, Phipson B, Wu D, Hu Y, Law CW, Shi W, Smyth GK (2015). limma powers differential expression analyses for RNA-sequencing and microarray studies. Nucleic Acids Res.

RETRACTED

[17] Gaujoux R, Seoighe C (2010). A flexible R package for nonnegative matrix factorization. BMC Bioinformatics.

[18] Kim H, Park H (2007). Sparse non-negative matrix factorizations via alternating non-negativity-constrained least squares for microarray data analysis. Bioinformatics.

[19] Zhang B, Horvath S (2005). A general framework for weighted gene co-expression network analysis. Stat Appl Genet Mol Biol.

[20] Zhang X, Feng H, Li Z, Li D, Liu S, Huang H, Li M (2018). Application of weighted gene co-expression network analysis to identify key modules and hub genes in oral squamous cell carcinoma tumorigenesis. Onco Targets Ther.

[21] Zhang X, Ren L, Yan X, Shan Y, Liu L, Zhou J, Kuang Q, Li M, Long H, Lai W (2020). Identification of immune-related lncRNAs in periodontitis reveals regulation network of gene-lncRNA-pathway-immunocyte. Int Immunopharmacol.

[22] Zeng D, Zhou R, Yu Y, Luo Y, Zhang J, Sun H, Bin J, Liao Y, Rao J, Zhang Y, Liao W (2018). Gene expression profiles for a prognostic immunoscore in gastric cancer. Br J Surg.

[23] Meyle J, Chapple I (2000). Molecular aspects of the pathogenesis of periodontitis. Periodontol.

[24] Jing L, Kim S, Sun L, Wang L, Mildner E, Divaris K, Jiao Y, Offenbacher S (2019). IL-37- and IL-35/IL-37-producing plasma cells in chronic periodontitis. J Dent Res.

[25] Afar B, Engel D, Clark EA (1992). Activated lymphocyte subsets in adult periodontitis. J Periodontal Res.

[26] Pan W, Wang Q, Chen Q (2019). The cytokine network involved in the host immune response to periodontitis. Int J Oral Sci.

[27] Artese L, Simon MJ, Piattelli A, Ferrari DS, Cardoso LA, Faveri M, Onuma T, Piccirilli M, Perrotti V, Shibli JA (2011). Immunohistochemical analysis of inflammatory infiltrate in aggressive and chronic periodontitis: a comparative study. Clin Oral Investig.

[28] Wang Q, Li M, Yang M, Yang Y, Song F, Zhang W, Li X, Chen K (2020). Analysis of immune-related signatures of lung adenocarcinoma identified two distinct subtypes: implications for immune checkpoint blockade therapy. Aging.

[29] Li Y, Xiao J, Bai J, Tian Y, Qu Y, Chen X, Wang Q, Li X, Zhang Y, Xu J (2019). Molecular characterization and clinical relevance of m(6)A regulators across 33 cancer types. Mol Cancer.

[30] Yang H, Zhang Q, Xu M, Wang L, Chen X, Feng Y, Li Y, Zhang X, Cui W, Jia X (2020). CCL2-CCR2 axis recruits tumor associated macrophages to induce immune evasion through PD-1 signaling in esophageal carcinogenesis. Mol Cancer.

[31] Otani Y, Yoo JY, Chao S, Liu J, Jaime-Ramirez AC, Lee TJ, Hurwitz B, Yan Y, Dai H, Glorioso JC (2020). Oncolytic HSV infected glioma cells activate NOTCH in adjacent tumor cells sensitizing tumors to gamma secretase inhibition. Clin Cancer Res.

RETRACTED

[32] Li Y, Ge D, Lu C (2019). The SMART App: an interactive web application for comprehensive DNA methylation analysis and visualization. Epigenetics Chromatin.

[33] Papalexi E, Satija R (2018). Single-cell RNA sequencing to explore immune cell heterogeneity. Nat Rev Immunol.

[34] Chen B, Khodadoust MS, Liu CL, Newman AM, Alizadeh AA (2018). Profiling tumor infiltrating immune cells with CIBERSORT. Methods Mol Biol.

[35] Finotello F, Trajanoski Z (2018). Quantifying tumor-infiltrating immune cells from transcriptomics data. Cancer Immunol Immunother.

[36] Yazdani S, Callemeyn J, Gazut S, Lerut E, de Loor H, Wevers M, Heylen L, Saison C, Koenig A, Thaunat O (2019). Natural killer cell infiltration is discriminative for antibody-mediated rejection and predicts outcome after kidney transplantation. Kidney Int.

[37] Panousis NI, Bertsias GK, Ongen H, Gergianaki I, Tektonidou MG, Trachana M, Romano-Palumbo L, Bielser D, Howald C, Pamfil C (2019). Combined genetic and transcriptome analysis of patients with SLE: distinct, targetable signatures for susceptibility and severity. Ann Rheum Dis.

[38] Liu R, Hu R, Zeng Y, Zhang W, Zhou HH (2020). Tumour immune cell infiltration and survival after platinum-based chemotherapy in high-grade serous ovarian cancer subtypes: A gene expression-based computational study. EBioMedicine.

